# LINC00311 promotes cancer stem‐like properties by targeting miR‐330‐5p/TLR4 pathway in human papillary thyroid cancer

**DOI:** 10.1002/cam4.2815

**Published:** 2020-01-02

**Authors:** Yu Gao, Fan Wang, Li Zhang, Mei Kang, Liyang Zhu, Lei Xu, Wei Liang, Wei Zhang

**Affiliations:** ^1^ Department of Radiotherapy The First Affiliated Hospital of Anhui Medical University Hefei Anhui China; ^2^ Department of Endocrinology Shengjing Hospital of China Medical University Shenyang Liaoning China

**Keywords:** LINC00311, MiR‐330‐5p, papillary thyroid cancer, spheroid formation, stem‐like properties, TLR4

## Abstract

Growing evidence has suggested that long noncoding RNAs (lncRNAs) play an essential role in the progression of papillary thyroid cancer (PTC). LncRNA LINC00311 was found to be able to regulate many cellular process in several diseases. However, the function and regulatory mechanism of LINC00311 remains unclear in PTC. In the present study, the results showed that the expression of LINC00311 was upregulated in PTC tissues and cells. Furthermore, knockdown of LINC00311 dramatically suppressed spheroid formation, proliferation, migration, and invasion in PTC cells in vitro. Mechanistic investigations revealed that LINC00311 was negatively correlated with the expression of miR‐330‐5p, meanwhile, TLR4 was a direct target of miR‐330‐5p. In addition, rescue assays further determined that LINC00311 contributed to the progression of PTC through regulating TLR4 expression. Taken together, these findings indicated that LINC00311 could promote cancer stem‐like properties by targeting miR‐330‐5p/TLR4 pathway in PTC.

## Graphical abstract

The expression of LINC00311 was increased in PTC tissues and cells, and knockdown of LINC00311 suppressed the spheroid formation in PTC cells,

## 1 INTRODUCTION

Thyroid cancer has gradually become one of the most malignant cancers over the past decades in the world.^1^ Among all types of thyroid tumors, papillary thyroid carcinoma (PTC) is the most common subtype of thyroid tumor with a good prognosis. In fact, the survival rate of this disease is extremely good.^2^, ^3^, ^4^ However, there are still 25% of PTC patients with predominant locoregional lymph node metastasis and recurrence, which may decrease the survival rate of PTC patients. In addition, the incidence of PTC is drastically increasing in recent years due to the improved diagnostic techniques over this time period.^5^, ^6^, ^7^, ^8^, ^9^ Therefore, it is essential to explore new and effective novel therapeutic targets for treating PTC.

Increasing evidence suggests that stem‐like properties of PTC cells play an essential role in the progression of different diseases, such as tumor metastasis, initiation, invasive growth, and so on.^10^ For example, Ahn et al^11^ showed that the percentage of CD44^+^/CD24^−^ cells was higher in aggressive recurrent PTC, meanwhile, as a stem cell marker, POU5F1 was found upregulated in the CD44^+^/CD24^−^ subpopulation and tumorigenic thyrospheroid cells. Further in clinical studies, stem cell markers have been found upregulated in PTC tissues, and the expression levels of these markers were positively correlated with lymph node, tumors metastasis stage.^12^ For treatment, one study suggested that PTC was more resistant to bortezomib, taxol, cisplatin, etoposide, and other chemotherapeutics drugs.^13^ In addition, another study reported that the expression of CD15, CD44, CD166, and ALDH1 was positively independently correlated with a shorter progression‐free survival (PFS).^14^ All these studies indicated that the stem‐like properties of PTC cells are not only closely related to the progression of PTC but also act as predictors for PTC prognosis. However, the molecular mechanism of stem‐like properties of PTC cells remains poorly understood.

Numerous studies have reported that, as members of noncoding RNAs (ncRNAs), microRNAs (miRNAs) and long noncoding RNAs (lncRNAs) play essential roles in regulating the pathologic network of PTC in different stages.^15^, ^16^, ^17^ LncRNAs are defined as a cluster of transcripts with more than 200 nucleotides without protein‐coding potential, which were originally considered as transcriptional noise. However, more and more evidence suggested that lncRNAs were involved in the regulation a wide range of cellular processes, and more importantly, play different roles in cancer stem‐like properties.^18^, ^19^, ^20^ For instance, lncRNA LUCAT1 plays an essential role in regulating breast cancer stemness.^21^ Another lncRNA NEAT1 has been shown to promote stem‐like properties in glioma cells.^22^ In addition, microRNAs (miRNAs) are defined as small, noncoding RNAs, which are approximately 21 nucleotides long and are able to repress translation or degradation of mRNA.^23^, ^24^ Accumulating evidences have proved that lncRNAs and miRNAs were abnormally expressed in PTC and can be used to determine the outcomes of PTC patients.^25^, ^26^, ^27^, ^28^ Recent studies reported that lncRNA LINC00311 participates in the process of cell proliferation and differentiation.^29^, ^30^ However, it is still unclear whether certain lncRNAs contribute to stem‐like properties in PTC cells.

In this study, we aimed to investigate the biologic function of lncRNA LINC00311 in PTC. Furthermore, we also want to clarify the related miRNA and the related pathways involved in stem‐like properties in PTC cells. These findings may provide a novel sight into the pathologic mechanism of PTC and might provide new therapeutic strategies.

## 2 MATERIALS AND METHODS

### 2.1 Collection and analysis of tumor tissues

The study was approved and supervised by the Ethical Committee of The First Affiliated Hospital of Anhui Medical University (Approval no. PJ2019‐04‐08) and all patients have signed the informed consents before any research‐related medical procedure. A total of 60 patients diagnosed with PTC were included in this study. For the subtype of PTC, 56 patients were diagnosed with conventional PTC, two of them were follicular variant of PTC, one was all cell variant of PTC, and one was confirmed as columnar cell variant of PTC. Sixty paired tissues (tumor and adjacent nontumor) were collected from patients who underwent surgical resection at The First Affiliated Hospital of Anhui Medical University. Chemotherapy or radiotherapy was not performed in those patients who were included in the current study. The definition of high or low expression of LINC00311 was determined by median. All samples were immediately snap‐frozen in liquid nitrogen and stored at −80°C for further studies.

### 2.2 qRT‐PCR

Total RNAs from samples (tissues and cells) were extracted by the Trizol reagents (Invitrogen). Then, extracted RNA was reverse transcribed into complementary DNA (cDNA). For miR‐330‐5p, MicroRNA Reverse Transcription Kit (Takara Biotechnology) was used to perform reverse transcription. Then, qRT‐PCR was performed with SYBR Green Master Mix (Life Technologies) using 7500 Real‐Time PCR system (Applied Biosystems). The primers used in our experiments were deigned and purchased from Sangon Biotech, which were listed in Table 1. The internal controls for miR‐330‐5p and mRNAs were U6 and GAPDH, respectively. The 2^ΔΔ^ Ct method was used to calculate the expression levels.

**Table 1:** Primers used in the present study

Gene	Primer sequence
miR‐330‐5p	forward: 5′‐TTTGGCGATCACTGCCTCTC‐3′
	reverse: 5′‐CTCTCTGCAGGCCGTGTG‐3′
U6	forward: 5′‐CTCGCTTCGGCAGCACA‐3′
	reverse: 5′‐AACGCTTCACGAATTTGCGT‐3′
LINC00311	forward: 5′‐CGCTGCGTCCTAACCAAATG‐3′
	reverse: 5′‐AGCAGAGCCAAGATGCTCAG‐3′
ALDH1	forward: 5′‐CCCGTGGCGTACTATGGATG‐3′
	reverse: 5′‐CAGTGCAGGCCCTATCTTCC‐3′
CD44	forward: 5′‐AGCAACTGAGACAGCAACCA‐3
	reverse: 5′‐CGTACCAGCCATTTGTGTTGT‐3′
NANO	forward: 5′‐AGAGCGAGAAGTGCCAACTC‐3
	reverse: 5′‐ GAGCGACTCATGCTGTGACT‐3′
SOX2	forward: 5′‐CATGACCAACTCGCAGACCT‐3
	reverse: 5′‐CCAAAGGAGTCCAGCAGTGT‐3′
Oct4	forward: 5′‐CTCGGACCTGGATGAGCTTC‐3′
	reverse: 5′‐TCAAAATCCTCGCGTTGGGA‐3′
TLR4	forward: 5′‐GAAGACTGGGTGCGGAATGA‐3
	reverse: 5′‐GACTCTGGGGTTTACCAGCC‐3′
GAPDH	forward: 5'‐CCGGGAAACTGTGGCGTGATGG‐3' reverse: 5'‐AGGTGGAGGAGTGGGTGTCGCTGTT‐3'

### 2.3 Cell lines and culture

Human thyroid cell line (HTori‐3), PTC cell lines (KTC‐1, K1, SNU‐790, TPC‐1), and HEK293 cells were purchased from ATCC. Cells were cultured in a standard humidified incubator with 95% air and 5% CO_2_ at 37°C. Cells were cultured in DMEM (Invitrogen) supplemented with 10% Fetal bovine serum (FBS) (Gibco), and 1% streptomycin/penicillin (100 μg/mL and 100 μg/mL) (Invitrogen).

### 2.4 Cell transfection

For transfection, short hairpin RNA (shRNA) plasmids targeting LINC00311 (sh1#‐ LINC00311, sh2#‐ LINC00311) and negative control (shNC), plasmid pcDNA3.1 TLR4 for overexpression of TLR4 and control vector, miR‐330‐5p mimic for overexpression of miR‐330‐5p and mimic control (NC mimics), miR‐330‐5p inhibitor for knockdown of miR‐330‐5p were purchased from Thermo Fisher scientific company. Different groups of cells were transfected using Lipofectamine 3000 (Invitrogen).

### 2.5 Immunohistochemistry (IHC)

The expression of TLR4, Ki67, and ALDH1 were detected by immunohistochemistry (IHC). Briefly, tissues were collected and fixed in 10% formaldehyde, then, each section was cut into 4 μm. Next, endogenous peroxidases were blocked with 3% H_2_O_2_ solution for avoiding nonspecific binding of primary antibodies. Then, those sections were incubated with primary anti‐TLR4 antibody (ab13556, 1:500, Abcam), anti‐Ki67 (ab15580, 1:1000, Abcam), and anti‐ALDH1 (ab56777, 1:1000, Abcam) at 4°C overnight. The following day, the secondary antibodies were added and incubated with sections for 1 hour at room temperature, and then the sections were immunostained using DAB plus kit. The images were then captured and analyzed.

### 2.6 Flow cytometer assay

The percentage of ALDH^+^ cells was determined by flow cytometry assay. Briefly, transfected TPC‐1 cells were resuspended in PBS at a density of 1 × 10^6^ cells and incubated in 1 mL of 5% BSA in phosphate buffer saline (PBS) for 1 hour. Then, approximately 100 μL of each cell suspension was incubated with 1 μL of ALDH^+^ antibody at 2‐8°C overnight. Cells were washed with 1 mL of 5% BSA in PBS and then the percentage of ALDH^+^ cells was measured and analyzed by flow cytometer.

### 2.7 Western blot assay

Total proteins from different groups of PTC cells were extracted by RIPA lysis buffer (Beyotime) and qualified by a BCA detection kit (Sigma). Subsequently, proteins were separated by sodium dodecyl sulfate‐polyacrylamide gel electrophoresis (SDS‐PAGE) and then transferred onto polyvinylidene fluoride (PVDF, Millipore) membranes. Primary antibodies suck as rabbit anti‐ALDH1 (ab52492, 1:500, Abcam), rabbit anti‐CD44 (ab216647, 1:1000, Abcam), rabbit anti‐NANOG (ab109250, 1:500, Abcam), rabbit anti‐SOX2 (ab97959, 1:500, Abcam), rabbit anti‐Oct4 (ab18976, 1:1000, Abcam), rabbit anti‐TLR4 (ab13556, 1:1000, Abcam), and β‐actin (ab8226, 1:1000, Abcam) were incubated with membranes at 4°C overnight after blocked in 5% nonfat milk. On the next day, the membranes were washed and then incubated with Goat Anti‐Rabbit secondary detection antibodies (1:4000; ab205718; Abcam). The protein of interest was detected using the LI‐COR Odyssey infrared imaging system (LI‐COR Bioscience).

### 2.8 Spheroid formation test

For spheroid formation test, different groups of transfected SNU‐790 and TPC‐1 cells, which have a density of 3.5 × 10^4^/well, were cultured in an Ultra‐Low Cluster plate (Costar). After 24 days, cells were stained with Crystal Violet, spheroids were photographed, and their diameter was calculated.

### 2.9 CCK‐8 assay

To assess the cell viability of PTC cells, CCK‐8 assays (ab228554, Abcam) were conducted. Briefly, different groups of PTC cells (3 × 10^3^) were seeded into 96‐well plates. After 48 hour, 10‐μL CCK‐8 reagent and 90‐μL DMEM were added to each well. Subsequently, cell absorbance was measured at a wavelength of 450 nm, 2 hours after incubation.

### 2.10 Colony formation

Colony formation assay was conducted in different groups. SNU‐790 and TPC‐1 cells were trypsinized and cultured in 6‐well plates. After 2 weeks, colonies were fixed with 10% (w/v) formaldehyde followed by 0.1% (w/v) crystal violet staining for 20 minutes. The colonies were photographed by a microscope (AF6000, Leica, Germany).

### 2.11 Wound healing

For wound healing assay, the cell monolayer was scratched using a 10‐μL pipette Eppendorf tip and then washed three times with PBS. After 24 hours, the percentage of wound closure was calculated by the following formula: Original width‐width after migration/Original width.

### 2.12 Transwell assay

Transwell assay was carried out using transwell chambers (Corning). A number of 5 × 10^3^ cells were seeded into the upper layer in basal medium without FBS, while lower chamber was filled with DMEM containing 10% FBS. The invaded cells were fixed and calculated after 24 hours.

### 2.13 Dual‐luciferase reporter assay

The 3′‐untranslated region (3′‐UTR) of LINC00311 was cloned into the pmirGLO vector (Promega) and named wild‐type (WT) LINC00311‐3′‐UTR. In addition, the fragments from TLR4 3′UTR containing the predicted miR‐330‐5p binding site or the corresponding mutants created by mutating the miR‐330‐5p seed region binding site were subcloned into the pmiRGLO Vector (Promega). Lipofectamine 2000 (Invitrogen) was used for transfection according to the manufacturer's protocol.

### 2.14 In situ hybridization (ISH)

Paraformaldehyde‐fixed, paraffin‐embedded PTC tissues were sectioned in 5‐μm thick, then sections were first stained to identify the tumor areas. The tissue microarray (TMA) consisted of triplicate 0.6‐mm cores using manual tissue microarrayer (Beecher Instruments). For normal control, we used adjacent histologically normal thyroid tissue.

For ISH test, LINC00311 was labeled with digoxin‐labeled RNA probe (BOSTER). The probes used were hs‐ LINC00311, hs‐ACTB (Actin, positive control), and dapB (negative control). Then, TMA was hybridized with LINC00311 probe overnight, followed by incubation with antibody against digoxigenin. Afterward, the signal was determined by diaminobenzidine (DAB) solution.

### 2.15 Fluorescence in situ hybridization (FISH)

Fluorescence In Situ Hybridization Kit (GenePharma) was used to perform FISH assay. LINC00311 and miR‐330‐5p were labeled with digoxin‐labeled RNA probe (red) and FAM probe (green). Hybridization was conducted at 55°C for 2 hours before the slides were washed and dehydrated. Afterward, air‐dried slides were then mounted with Prolong Gold Antifade Reagent with DAPI (blue). Images were captured using Leica SP8 laser scanning confocal microscope.

### 2.16 RIP

Magna RIP™ RNA‐Binding Protein Immunoprecipitation Kit (Millipore) was applied in our study to identify the binding relationship between endogenous LINC00311 and miR‐330‐5p. The cell lysates were incubated in a RIP buffer containing the magnetic beads, which had been coated with Ago2 antibodies or negative control IgG. Then, the precipitation of RNA was isolated and analyzed.

### 2.17 Tumor xenograft experiments

The animal procedures were approved by the Ethical Committee of The First Affiliated Hospital of Anhui Medical University (Approval no. LLSC20190721). Six 6‐ to 8‐week‐old BALB/c nude mice were purchased from Charles River. For tumorigenesis experiments, TPC‐1 cells, which transfected with sh‐LINC00311 or shNC, were subcutaneously inoculated into the right flanks of mice (0 day). Tumor volume was monitored and measured every 4 days. The nude mice were sacrificed after 24 days, and the weight of each tumor was measured. In addition, the tumor tissue was collected for further experiments.

### 2.18 Statistical analysis

All data were presented as Mean ± SD of three independent experiments and analyzed using SPSS v19.0 and GraphPad Prism 7. All cell experiments were independently repeated at least in triplicate. For comparing two groups or multiple groups, Student's *t* test and one‐way ANOVA were used, respectively. Survival curves were determined by Kaplan‐Meier analysis. Furthermore, Pearson correlation coefficient and Kaplan‐Meier analysis were used for analyzing statistical correlation and survival curves, respectively. *P* values (*P < .05; **P < .01) less than 0.05 or 0.01 considered statistically significant.

## 3 RESULTS

### 3.1 The expression of LINC00311 was increased in PTC tissues and cells

In order to identity the expression of LINC00311 in human PTC tissues, 60 pairs of PTC and adjacent normal tissues were included and analyzed. Figure 1A showed that the expression of LINC00311 was significantly upregulated in PTC tissues compared with normal tissues (*P* < .01). In addition, in tumor tissues, the definition of high or low expression of LINC00311 was determined by median, which means, it was relatively highly expressed in 30 PTC tissues, whereas it was relatively lower expressed in another 30 PTC tissues. Moreover, in ISH test, at both 40× and 100× magnifications, moderate to strong signals of LINC00311 expression were observed in PTC tissues. The results revealed that LINC00311 was upregulated in PTC tissues. In addition, the correlation between LINC00311 expression and clinicopathological characteristics of PTC patients was analyzed (Table 2). The high level of LINC00311 was positively correlated with advanced primary tumor (T3‐T4), lymph node metastasis (N1) as well as TNM stage (III‐IV) in PTC patients (*P* < .05, Table 2). Moreover, Kaplan‐Meier analysis showed that the high level of LINC00311 was correlated with poor overall survival in PTC patients (*P* = .0352, Figure 1C). In addition, the expression of LINC00311 was detected both in human thyroid cell line (HTori‐3) and PTC cell lines (KTC‐1, K1, SNU‐790, TPC‐1) using qRT‐PCR. As shown in Figure 1D, our results demonstrated that LINC00311 was markedly upregulated in all PTC cell lines compared with normal human thyroid cell, especially in SNU‐790 and TPC‐1 cell lines (*P* < .01). We further measured the expression of LINC00311 in monolayer and spheroid cells, respectively. Compared with monolayer cells, the expression of LINC00311 was higher in spheroid cells, suggesting that LINC00311 was mainly expressed in spheroid PTC cells (*P* < .01, Figure 1E). Taken together, these results reveled that LINC00311 was upregulated in PTC tissue and cell lines and correlated with lower overall survival and worse outcome in PTC patients.

**Figure 1:** The highly expressed LINC00311 was associated with poor clinical outcome of papillary thyroid cancer (PTC) patients. A, Relative expression of LINC00311 in PTC tissues and paired normal tissues was analyzed using qRT‐PCR. B, The expression of LINC00311 was detected in PTC tissues and paired normal tissues using FISH test. C, Kaplan‐Meier analysis exhibited the survival rate of PTC patients with high or low expression levels. D, The expression of LINC00311 was detected in human thyroid cell line (HTori‐3) and PTC cell lines (KTC‐1, K1, SNU‐790, TPC‐1) using qRT‐PCR. E, The expression of LINC00311 was analyzed in monolayer and spheroid PTC cells lines, respectively. Data were expressed as mean ± SD. **P < .01, ***P < .001 represent statistical difference

**Table 2:** Association between LINC00311 expression and clinicopathological characteristics of PTC patients

Parameters	LINC00311 expression		*P* value
	Low (n = 30)	High (n = 30)	
Gender			.605
Male	13	15	
Female	17	15	
Age (y)			.791
<45	11	12	
≥45	19	18	
Focality			.284
Unifocal	17	21	
Multifocal	13	9	
Extrathyroidal extension			.781
Positive	9	10	
Negative	21	20	
Primary tumor			.009*
T1‐T2	18	8	
T3‐T4	12	22	
Lymph node metastasis			.020*
N0	20	11	
N1	10	19	
TNM stage			.004*
I‐II	21	10	
III‐IV	9	20	

*P < .05 represent statistically difference.

### 3.2 Knockdown of LINC00311 attenuated spheroid formation in PTC cells

To assess the potential pathologic role of LINC00311 in PTC, loss‐of‐function experiments were conducted in our study. Firstly, knockdown efficiency of LINC00311 was tested in two knockdown systems (sh#1‐LINC00311, sh#2‐LINC00311) in ALDH^+^ SNU‐790 and TPC‐1 cell lines. Compared with control vector (shNC), the expression of LINC00311 was significantly inhibited in two cell lines in these two knockdown systems, indicating that the current method can be used for further studies (*P* < .01, Figure 2A). Then, the number of spheres and diameter of spheres were measured and analyzed. As shown in Figure 2B, the number of spheres was obviously suppressed by the knockdown of LINC00311 (*P* < .01), meanwhile, the diameter of spheres was also decreased in the LINC00311 knockdown group (*P* < .01). In addition, stemness markers, such as ALDH1, CD44, NANOG, SOX2, and Oct4, were detected in both mRNA level and protein level in PTC cells. The results revealed that knockdown of LINC00311 significantly suppressed the expression of these markers in both mRNA level and protein level (*P* < .01, Figure 2C,D). Furthermore, flow cytometry assay was used for analyzing relative percentage of ALDH^+^ cells in PTC cell lines. As shown in Figure 2E, the percentage of ALDH^+^ cell was markedly lower in LINC00311 knockdown groups compared with the vector group (*P* < .05, *P* < .01). Overall, these results demonstrated that knockdown of LINC00311 suppressed spheroid formation in PTC cells.

**Figure 2:** The expression of spheroid formation markers in LINC00311‐knockdown papillary thyroid cancer (PTC) cells. A, The expression level of LINC00311 was detected by qRT‐PCR in ALDH^+^ SNU‐790 and TPC‐1 cell lines transfected with shRNAs targeted LINC00311 (sh#1‐LINC00311, sh#2‐LINC00311). B, Number of spheres and diameter of spheres of PTC cells were measured and analyzed in LINC00311‐knockdown group and control group, respectively. The effect of downregulated LINC00311 on stemness markers such as ALDH1, CD44, NANOG, SOX2, and Oct4 was detected by qRT‐PCR (C) and Western blot (D). E, Flow cytometer assay was used for analyzing relative percentage of ALDH^+^ cells in different groups. Data were expressed as mean ± SD. *P < .05, **P < .01, ***P < .001 represent statistical difference

### 3.3 Knockdown of LINC00311 attenuated cell proliferation, migration, and invasion in PTC cells

Next, we investigated the functional roles of LINC00311 in PTC cells using knockdown system. Cell viability was measured by CCK‐8 assay. As shown in Figure 3A, after transfected with sh‐LINC00311, cell viability was inhibited in ALDH^+^ SNU‐790 and TPC‐1 cell lines (*P* < .05). Colony formation assay showed that knockdown of LINC00311 attenuates the colony number of ALDH^+^ SNU‐790 and TPC‐1 cells (*P* < .01, Figure 3B). Subsequently, wound healing assay and transwell assay were conducted to investigate the migration and invasion abilities of PTC cells. Our results demonstrated that cells transfected with sh‐LINC00311 showed a slower closing of scratch wound and less invasion cell numbers compared with control vector (shNC) in ALDH^+^ SNU‐790 and TPC‐1 cell lines, suggesting that knockdown of LINC00311 inhibited cell migration and invasion in PTC cells (*P* < .05, *P* < .01, Figure 3C,D). Altogether, the above results indicated that knockdown of LINC00311 suppressed cell proliferation, migration, and invasion in PTC cells.

**Figure 3:** LINC00311 knockdown inhibited cell proliferation, migration, and invasion in papillary thyroid cancer (PTC) cells. A, Cell viability was detected by CCK‐8 assay in different groups (sh#1‐LINC00311, sh#2‐LINC00311, and shNC). B, The role of knockdown of LINC00311 on cell proliferation was determined by colony formation assay. C, The effect of downregulated LINC00311 on migration ability in PTC cells (ALDH^+^ SNU‐790 and TPC‐1) was measured by wound healing assay. D, Transwell assay was used to detect the invasion of PTC cells (ALDH^+^ SNU‐790 and TPC‐1) in different groups (sh#1‐LINC00311, sh#2‐LINC00311, and shNC). Data were expressed as mean ± SD. *P < .05, **P < .01 represent statistical difference

### 3.4 The expression of LINC00311 was negatively correlated with the expression of miR‐330‐5p

To better explore the underlying molecular mechanisms of the effects of LINC00311 on PTC cellular behavior, we conducted bioinformatics analysis via miRDB. We found a putative miR‐330‐5p response elements on LINC00311 (Figure 4A). Then, FISH assay revealed that LINC00311 and miR‐330‐5p were all expressed in the cytoplasm of PTC cells (Figure 4B). Next, qRT‐PCR was used for testing the transfection efficiency of miR‐330‐5p overexpression. As shown in Figure 4C, after transfected with miR‐330‐5p mimic, the expression of miR‐330‐5p was markedly increased compared with control miR‐NC mimic (*P* < .01, Figure 4C). Subsequently, dual‐luciferase reporter assay was conducted to confirm the targeting relationship between LINC00311 and miR‐330‐5p. As shown in Figure 4D, luciferase activity of HEK 293 cells transfected with LINC00311 WT plasmid was significantly inhibited by miR‐330‐5p mimics (*P* < .01), indicating that miR‐330‐5p can bind to LINC00311. In addition, RIP assay results suggested that compared with IgG control, LINC00311 preferentially enriches the miRNA ribonucleoprotein complex containing Ago2 (*P* < .01, Figure 4E). Moreover, the expression of miR‐330‐5p was significantly increased in PTC cells transfected with sh‐LINC00311 (*P* < .01, Figure 4F). Furthermore, in tumor samples, the expression level of miR‐330‐5p was much lower than normal tissues (*P* < .05, Figure 4G). By using Spearman's correlation analysis, the expression of LINC00311 and miR‐330‐5p exhibited a dramatical negative correlation, which was shown in Figure 4H (*P* < .001, r = 0.7723). All these data demonstrated that the expression of LINC00311 was negatively correlated with miR‐330‐5p.

**Figure 4:** LINC00311 inversely interacted with miR‐330‐5p. A, LINC00311 wide‐type and the mutated‐type in the miR‐330‐5p binding sites were shown. B, The co‐localization of LINC00311 and miR‐330‐5p was tested using FISH assay. C, The transfection efficiency of miR‐330‐5p mimics was tested by qRT‐PCR. D, Luciferase activity of HEK293 cells co‐transfected with miR‐330‐5p mimics or NC mimics and luciferase reporters containing LINC00311 WT or LINC00311 MUT transcript were determined by dual‐luciferase reporter assays. E, Endogenous miR‐330‐5p precipitated by AGO2 upon overexpression of LINC00311 was determined by RIP assay. F, The expression of miR‐330‐5p was measured by qRT‐PCR in different groups. G, The expression of miR‐330‐5p in papillary thyroid cancer (PTC) tissues and corresponding normal tissues was detected by qRT‐PCR. n = 60. H, The correlation between LINC00311 and miR‐330‐5p was analyzed using Spearman's correlation analysis. Data were expressed as mean ± SD. *P < .05, **P < .01 represent statistical difference

### 3.5 TLR4 was a direct target of miR‐330‐5p

Subsequently, the role of miR‐330‐5p and its function in the pathogenesis of PTC were further explored. Among the putative targets, we focused on TLR4, which mediates the expression of a variety of genes in response to various cell functions. Figure 5A showed the biding site of TLR4 and miR‐330‐5p. We further conducted luciferase reporter assay by co‐transfection of miR‐330‐5p mimics or NC mimics and TLR4 3′‐UTR WT or TLR4 3′‐UTR MUT transcript into HEK293 cells. The results indicated that TLR4 was a target gene of miR‐330‐3p (*P* < .01, Figure 5B). Then, the transfection efficiency of miR‐330‐5p inhibitor was examined. As shown in Figure 5C, after transfected with miR‐330‐5p inhibitor, the expression of miR‐330‐5p was dramatically inhibited by its inhibitor in ALDH^+^ SNU‐790 and TPC‐1 cells (*P* < .01). Then, the expression of mRNA and protein level of TLR4 were detected by qRT‐PCR. The results showed that the expression of TLR4 mRNA and TLR4 protein was significantly increased when cells were transfected with miR‐330‐5p inhibitor (*P* < .01, Figure 5D,E). On the contrary, TLR4 was decreased when cells were transfected with miR‐330‐5p mimics (*P* < .01, Figure 5D,E), indicating that the expression of TLR4 was negatively related with miR‐330‐5p in ALDH^+^ SNU‐790 and TPC‐1 cells. Moreover, the expression of TLR4 mRNA was detected in human PTC tissues and normal tissues (n = 60). The results demonstrated that mRNA level of TLR4 was significantly upregulated in tumor tissues compared with nontumor tissues (*P* < .01, Figure 5F). This result was further confirmed by IHC staining (Figure 5G). In addition, the correlation between TLR4 and LINC00311 and TLR4 and miR‐330‐5p was analyzed, and the results suggested that the expression of TLR4 was positively correlated with LINC00311 level (r = 0.7577, *P* < .001), while negatively correlated with miR‐330‐3p (r = −0.6072, *P* < .001, Figure 5H). Taken together, these results indicated that TLR4 was a direct target of miR‐330‐5p.

**Figure 5:** TLR4 was a direct target of miR‐330‐5p. A, Biding site of TLR4 and miR‐330‐5p was shown. B, Luciferase activity of HEK293 cells co‐transfected with miR‐330‐5p mimics or NC mimics and luciferase reporters containing TLR4 WT or TLR4 MUT transcript were determined by dual‐luciferase reporter assays. C, The transfection efficiency of miR‐330‐5p inhibitors was tested by qRT‐PCR. D, The expression of mRNA TLR4 was detected in papillary thyroid cancer (PTC) cells, which transfected with miR‐330‐5p mimic, inhibitor, miR‐NC, and inhi‐NC, using qRT‐PCR. E, The expression of TLR4 protein was detected in PTC cells, which transfected with miR‐330‐5p mimic, inhibitor, miR‐NC, and inhi‐NC, using Western blot. F, The expression of TLR4 in PTC tissues and corresponding normal tissues was detected by qRT‐PCR. n = 60. G, The expression of TLR4 was measured in tumor and normal tissues using IHC. H, The correlation between TLR4 and LINC00311 or miR‐330‐5p was analyzed using Spearman's correlation analysis. Data were expressed as mean ± SD. *P < .05, **P < .01 represent statistical difference

### 3.6 LINC00311 promotes stem‐like properties in PTC cell lines via targeting TLR4

Given the fact that LINC00311 was directly interacted with miR‐330‐5p while TLR4 was a direct target of miR‐330‐5p, we hypothesized that LINC00311 might exert its role in regulating PTC cellar functions via targeting TLR4. To this end, we used TLR4 overexpression plasmid pcDNA3.1‐TLR4, and the level of TLR4 mRNA and TLR4 protein was significantly increased in ALDH^+^ TPC‐1 cells transfected with pcDNA3.1‐TLR4 (*P* < .01, Figure 6A,B). Next, to test whether LINC00311 is able to promote stem‐like properties in PTC cell lines via targeting TLR4, ALDH^+^ TPC‐1 cells were co‐transfected with sh‐LINC00311 or shNC and pcDNA3.1‐TLR4 or control vector. Then, the number and diameter of spheres, stemness markers, and percentage of ALDH^+^ cells were detected in different groups, respectively. The results demonstrated that compared to control, interference of LINC00311 markedly inhibited the number and diameter of spheres, expression of stemness markers such as ALDH1, CD44, NANOG, SOX2, and Oct4, as well as percentage of ALDH^+^ cells (*P* < .05, *P* < .01, Figure 6C‐E). However, these effects were reversed by the overexpression of TLR4 (*P* < .01, Figure 6C‐E). Moreover, cell viability, proliferation, migration, and invasion abilities were detected using CCK‐8 assay, colony formation assay, wound healing assay, and transwell assay, respectively. As shown in Figure 6F‐I, overexpression of TLR4 abolished the INC00311‐induced effects on cell viability, proliferation, migration, and invasion (*P* < .05, *P* < .01). Collectively, the data indicated that LINC00311 promoted stem‐like properties in PTC cell lines via targeting TLR4.

**Figure 6:** LINC00311 promotes stem‐like properties in papillary thyroid cancer (PTC) cell lines via targeting TLR4. A‐B, The transfection efficiency of pcDNA3.1‐TLR4 was tested by qRT‐PCR and Western blot, respectively. C, Number of spheres and diameter of spheres of ALDH^+^ TPC‐1 cells transfected with co‐transfected with sh‐LINC00311 or shNC and pcDNA3.1‐TLR4 or control vector were measured and analyzed. D, Stemness markers such as ALDH1, CD44, NANOG, SOX2, and Oct4 were detected by Western blot in different groups. E, Flow cytometer assay was used for analyzing relative percentage of ALDH^+^ TPC‐1 cells in different groups. F‐I, The cell viability, proliferation, migration, and invasion were determined by CCK‐8 assay, colony formation assay, wound healing assay, and transwell assay in ALDH^+^ TPC‐1 cells, which were co‐transfected with sh‐LINC00311 or shNC and pcDNA3.1‐TLR4 or control vector. Data were expressed as mean ± SD. *P < .05, **P < .01 represent statistical difference

### 3.7 Knockdown of LINC00311 suppressed PTC cell tumorigenesis in vivo

In the final part, orthotopic xenograft mouse models were used to identify the effect of LINC00311 on PTC in vivo. ALDH^+^ TPC‐1 cells transfected with shRNA LINC00311 or control plasmid (shNC) were inoculated into nude mice (n = 6). First, the transfection efficiency of shRNA LINC00311 was tested in ALDH^+^ TPC‐1 cells. The results showed that the expression of LINC00311 and mRNA TLR4 was markedly downregulated, while the expression of miR‐330‐5p was significantly increased when transfected with shRNA LINC00311 compared with shNC (*P* < .01, Figure 7A). Then, tumor volume and tumor weight were measured 24 days after initial inoculation. As shown in Figure 7B,C, the tumor volume and weight were dramatically reduced in shRNA LINC00311‐treated group compared with control group (*P* < .05, *P* < .01). Furthermore, the expression of TLR4, Ki67 (proliferative marker), and ALDH1 (stemness marker) was detected by IHC assay. Compared with control, the expression of TLR4, Ki67, and ALDH1 was relatively lower in shRNA LINC00311 group (Figure 7D). All results revealed that knockdown of LINC00311 suppressed PTC cell tumorigenesis in vivo.

**Figure 7:** Downregulated LINC00311 expression suppressed PTC cell tumorigenesis in vivo. A, The expression of LINC00311, miR‐330‐5p, and TLR4 was measured in ALDH^+^ TPC‐1 cells after transfected with sh‐LINC00311 or shNC. B, Tumors collected from mice, which received ALDH^+^ TPC‐1 cell inoculation (sh‐LINC00311 or shNC), were shown. C, Tumor volume and weight were detected after initial subcutaneously inoculation in nude mice. n = 6. D, The expression level of TLR4, proliferation indicator Ki67, stemness marker ALDH1 in vivo was detected by IHC assay. Data were expressed as mean ± SD. *P < .05, **P < .01 represent statistical difference

## 4 DISCUSSION

With the increasing incidence and limited therapeutic targets, PTC has attracted much more attention in the past few decades.^31^ Clinically, identifying accurate molecular markers for targeting PTC is critically essential in the early stage of PTC, as some of the patients have risk of distal metastasis.^32^ Recently, considerable evidence suggested that lncRNAs play various roles in biological process of PTC. For instance, lncRNA TUG1 contributes to the progression of PTC by regulating miR‐145.^33^ Another lncRNA called ABHD11‐AS1 was dramatically upregulated in PTC cells and promoted tumorigenesis via modulating BHD11‐AS1/miR‐199a‐5p/SLC1A5 axis.^33^ In addition, lncRNA myocardial infarction‐associated transcript (MIAT) was also highly expressed in PTC cells and enhanced tumor progression.^34^, ^35^ From our perspective, most of the reported lncRNAs were abnormally upregulated in PTC samples and cells and have negative impact on outcome of PTC patients. For the cellular and molecular mechanisms, these lncRNAs may closely associated with some cell functions such as proliferation, migration, apoptosis, and invasion by regulating numerous signaling pathways.^36^, ^37^, ^38^ In this study, we focused on a new lncRNA called LINC00311, which was previously reported to be highly expressed in osteoclasts and elevated the expression Notch2 and TRAP mRNA.^22^ Our results showed that LINC00311 was also upregulated in human PTC tissue and cell lines. Furthermore, by conducting a series of loss‐of‐function experiments, we found that the knockdown of LINC00311 inhibited spheroid formation, proliferation, migration, and invasion in PTC cells in vitro, suggesting that LINC00311 indeed play a regulatory role in PTC pathologic process. In addition, higher expression of LINC00311 in PTC tissues was correlated with poor outcome of PTC.

Stem‐like cells are defined as a subpopulation of self‐renewing stem cells, which are more resistant to chemotherapeutics or radiation therapy.^39^ To date, accumulating evidence from advances in tumor cell biology and genetics have suggested that stem‐like properties in cell play a critical role in tumor initiation, invasive growth, and metastasis in many cancers.^40^, ^41^ In PTC cell lines, especially in stem‐like properties population, the most putative cancer stem cell markers are CD44, ALDH1, NANOG, etc^42^, ^43^ In addition, studies have reported that some lncRNAs, such as lncRNA‐H19, were specifically highly expressed in PTC stem cells, meanwhile, silencing of H19 suppressed E2‐induced sphere formation ability,^44^ indicating that in PTC, certain lncRNAs may be involved in cell stemness ability. In this study, the expression of stemness markers, such as ALDH1, CD44, NANOG, SOX2, and Oct4, was detected in both mRNA level and protein level in LINC00311 knockdown group or control group, as previously described. The results showed that LINC00311 significantly suppressed the expression of these markers, suggesting that knockdown of LINC00311 suppressed spheroid formation and stemness in PTC cells.

To further investigate the molecular mechanism of how LINC00311 exerts its function in PTC stem‐like properties, we used bioinformatics tools to predict its potential target. By using dual‐luciferase reporter assay, RIP, and qRT‐PCR, we found that the level of LINC00311 was negatively correlated with miR‐330‐5p. Moreover, toll‐like receptors 4 (TLR4) was a direct target of miR‐330‐5p. As important downstream factors of LINC00311 in our study, miR‐330‐5p and TLR4 were also confirmed involved in cancer pathological progressions in many published studies. So far, miR‐330‐5 was reported as an inhibitory factor in many types of cancers, such as glioblastoma,^45^ cutaneous malignant melanoma,^46^ and ovarian cancer.^47^ However, until now, no studies have reported the miR‐330‐5p in PTC yet. TLR4 was abundantly expressed in PTC cells and PTC.^48^ Moreover, overexpression of TLR4 induces ETS1 transcriptional activity by regulating MAPK/ERK pathway.^49^ Our study demonstrated that LINC00311 promotes stem‐like properties in PTC cell lines via targeting TLR4, indicating that TLR4 was interacted with LINC00311 in the pathologic process in PTC progression. However, there are still some limitations in the current study. For example, we did not introduce miR‐330‐5p knockdown or overexpression system into the functional experiments. Moreover, we did not design any experiments to clarify whether off‐target effects of shRNA exist or not in the current experiments. Additionally, only the loss‐of‐function experiments were performed in the present study, gain‐of‐function studies may also need to valid the results in future.

In summary, our studies revealed that lncRNA LINC00311 played a regulator role in promoting PTC stem‐like traits. In addition, LINC00311 accelerated this process via modulating miR‐330‐5p/TLR4 pathway. The current findings may provide a better understanding of molecular mechanism of PTC cell stemness, and may further contribute to a potential therapeutic opportunity for aggressive PTC.

## CONFLICT OF INTEREST

The authors declare that they have no competing interests, and all authors should confirm its accuracy.

## AUTHOR CONTRIBUTIONS

WZ and YG conceived and designed the experiments, FW, LZ, and MK analyzed and interpreted the results of the experiments, LYZ, LX and WL performed the experiments.

## ETHICS APPROVAL AND CONSENT TO PARTICIPATE

All procedures performed in studies involving human participants were in accordance with the standards upheld by the Ethics Committee of Shengjing Hospital of China Medical University and with those of the 1964 Helsinki Declaration and its later amendments for ethical research involving human subjects. (Approval No. 20190721).

All animal experiments were approved by the Ethics Committee of Shengjing Hospital of China Medical University for the use of animals and conducted in accordance with the National Institutes of Health Laboratory Animal Care and Use Guidelines. (Approval No. PJ‐2019‐04‐08).

## INFORMED CONSENT

Written informed consent was obtained from a legally authorized representative(s) for anonymized patient information to be published in this article.

## Data Availability

All data generated or analyzed during this study are included in this published article.
